# Assessment of Salivary Mutans Streptococci Counts to Atraumatic Restorative Treatment Among Children: A Randomised Controlled Trial

**DOI:** 10.7759/cureus.32126

**Published:** 2022-12-02

**Authors:** Milind Wasnik, Abhishek Sharma, Harsh G Shah, Vasudha Sodani, Ajithkrishnan CG

**Affiliations:** 1 Department of Public Health Dentistry, Government Dental College & Hospital, Raipur, IND; 2 Department of Public Health Dentistry, Government Dental College & Hospital, Jaipur, IND; 3 Department of Public Health Dentistry, Ahmedabad Dental College & Hospital, Ahmedabad, IND; 4 Department of Pedodontics & Pediatric Dentistry, Ahmedabad Dental College & Hospital, Ahmedabad, IND; 5 Department of Public Health Dentistry, K M Shah Dental College & Hospital, Vadodara, IND

**Keywords:** art, streptococcus mutans, atraumatic restoration, glass-ionomer cement, colony-forming units

## Abstract

Introduction

Besides the survival rate of restorations, the effect of atraumatic restorative treatment (ART) on bacterial count is also important. After ART restoration, the bacterial count drops due to the fluoride's antibacterial activity and hence it can decrease the chances of further decay. The present study assessed salivary mutans streptococci counts for six months of evaluations subsequent to ART among 12-15-year-old children attending schools in Piparia village, Vadodara district.

Methods

ART was performed on 32 children and followed up after six months to evaluate the success rate of ART. Saliva collection and microbial analysis were performed five times from every participant, before ART restoration placement, seven days, 30 days (one month), 90 days (three months) and 180 days (six months) post-restoration.

Results

At baseline, the mean colony forming units (CFU) was 48.30 ± 46.58, which reduced to 32.64 ± 30.40 at one week, which showed a 32% reduction in colony counts. This further reduced to 18.60 ± 20.81 at one month, marking a further 43% reduction in colony counts. This again reduced to 13.63 ± 18.04 at three months, which showed a 27% reduction in colony counts. CFU came to 16.23 ± 23.34 at six months, which showed a 19% increase in colony counts. Comparison of baseline mean CFU (48.30 ± 46.58) to six months mean CFU of streptococcus mutans (SM) (16.23 ± 23.34) showed a 66% reduction in colony counts. A statistically significant difference was found between numerous intervals of time of CFU of streptococcus mutans.

Conclusion

The findings reveal that ART is a clinical treatment that can be used to treat caries in young children, and it helped significantly reduce Streptococcus Mutans levels in saliva.

## Introduction

Dental caries is a localized carbohydrate-modified infection that destroys a tooth's hard tissues, typically going beyond the reversible stage in many countries; many individuals assume that tooth loss is an inevitable part of life. At this stage, extraction is often the only treatment option. The World Health Organization (WHO) emphasizes the need to develop a new approach to dental care for use in economically underdeveloped areas. In the International Association of Dental Research (IADR) annual meeting of 1994, the WHO recognized, endorsed, and promoted atraumatic restorative treatment (ART) worldwide [1-3]. On 7th April 1994, the WHO, on the occasion of World Oral Health Day, launched the Manual of Atraumatic Restorative Treatment (ART) - Dental Caries Technique [4].

With hand instruments, the dentist in the ART approach excavates cavitated dentine caries, restores the cavity, and seals any related pits and fissures with an adhesive-filling substance. ART is considered a combined preventive and restorative procedure, resulting in sealant restoration. Besides the survival rate of the restoration, the effect of ART on bacterial count is also important. After ART restoration, the bacterial count drops due to the fluoride's antibacterial activity and hence it can decrease the chances of further decay. Only a few studies revealed a significant reduction in salivary Streptococcus mutans (SM) after ART restoration [5,6]. SM has all of the virulent characteristics needed to have a role in the caries process [7]. SM has been found in dentine in previous studies [8]. These are opportunistic pathogens that can be present as resident microflora in people who do not have caries and can become pathogenic when environmental conditions are appropriate.

In the literature review, it was evident that there is a scarcity of studies on the evaluation of salivary mutans streptococci count after ART amongst school-going children. Hence the present study was conducted to evaluate salivary mutans streptococci count after six months of performing ART amongst 12-15-year-old school-going children of Piparia village of Vadodara district, Gujarat, India.

## Materials and methods

A list of schools was obtained from the Gram Panchayat office in Piparia village, and only one was found to provide education from the fifth to the tenth standard. There were a total of 80 students aged between 12-15 years that were studying in the school. Out of these 80, 32 did not consent to be screened by us. Resultantly, we screened the remaining 48 school children who were willing to get oral health aged between 12-15 years, and 32 school children, out of which 18 (56.25%) were males and 14 (43.75%) females, were found to be suitable for our study’s objectives. Our study protocol was reviewed and approved by the Human Research Review Panel as well as the college ethics committee. After defining the study's objective, each participant's parent signed a written informed consent form indicating their willingness to participate in the study.

Only the students having one or more carious lesions involving dentine in permanent teeth, which is accessible to hand instruments and can be treated with ART, were included. All the children who did not consent to get screened were excluded from the domains of our study. The principal investigator conducted the study with the help of a trained assistant. ART was performed on 10 children at the Department of Public Health Dentistry under the supervision of a senior faculty member. The follow-up after six months was carried out for ART success rate evaluation according to the prescribed ART assessment criteria given by Frencken et al. (Table 1) [9].

**Table 1:** Atraumatic restorative treatment (ART) assessment criteria

Score	Criterion
0	Present, good
1	Present, a slight marginal defect for whatever reason, at any one place which is less than 0.5 mm in depth. No repair is needed.
2	Present, a marginal defect for whatever reason, at any one place which is deeper than 0.5 mm but less than 1.0 mm. Repair is needed.
3	Present, gross defect of more than 1.0 mm in depth. Repair is needed.
4	Not present, restoration has (almost) completely disappeared. Treatment is needed.
5	Not present, other restorative treatment has been performed.
6	Not present, the tooth has been extracted.
7	Present, wear and tear gradually over larger parts of the restoration but is less than 0.5 mm at the deepest point. No repair is needed.
8	Present, wear and tear gradually over larger parts of the restoration which is deeper than 0.5 mm. Repair is needed.
9	Unable to diagnose.

Saliva collection

Saliva collection and microbial analysis were performed five times for every participant, i.e., prior to ART restoration placement, seven days, 30 days (one month), 90 days (three months) and 180 days (six months) post-restoration. A 1-gram piece of unflavoured paraffin wax was given to each child and asked to chew for 1 minute. Two-millilitre of the whole saliva was collected into a saliva collecting chamber. A code number identified the saliva samples of all the patients during sample collection and processing. During subsequent saliva sample collection, the same code number was used for the same patient. Collected saliva was used to estimate the mutant’s streptococci level by using the dip slide method [10].

Microbial analysis

The saliva samples were vortexed before being used (15 sec, Cyclomixer, REMI CM 101, REMI Sales & Engineering Ltd., Goregaon (East), Mumbai, Maharashtra, India). With potassium tellurite medium, one loop (1/1000th ml of material) was infected on Mitis Salivarius Agar (Himedia M259, Lot No Y1100, HiMedia Laboratories Pvt. Ltd, Mumbai, Maharashtra, India). The plates were incubated for 48 hours at 37°C in a jar containing 5-10% CO2. The counts were made of colonies with morphologic characteristics of Streptococcus mutans (0.5 mm raised convex undulated colonies of light blue color with rough margins, granular frosted glass appearance) on the plates using a magnifying lens and were expressed as a number of colony-forming units (CFU) per/ml of saliva. Semi-quantitation of the number of colonies was done by multiplying the actual colony count with 1×10^3^ as the sample was diluted one thousand times (1:5 dilution).

Statistical analysis

The Statistical Package for Social Sciences (SPSS) for Windows 26.0 (IBM Corp., Armonk, NY) was used to enter and analyze the data. The 95% confidence interval was used, and a p-value of 0.05 was considered statistically significant. Descriptive statistics were applied for demographic details. Shapiro-Wilk test was used, and it showed that data was not parametric; hence Wilcoxon signed-rank test was used. Wilcoxon signed-rank test was used for comparing the mean colony forming units (CFU) at various time intervals.

## Results

Table 2 illustrates demographic information.

**Table 2:** Distribution of subjects according to age and gender

Age	Male (%)	Female (%)	Total (%)
12 Years	5 (55.55)	4 (44.45)	9 (100)
13 Years	5 (62.5)	3 (37.5)	8 (100)
14 Years	4 (57.14)	3 (42.86)	7 (100)
15 Years	4 (50)	4 (50)	8 (100)
Total	18 (56.25)	14 (43.75)	32 (100)

Out of 32 subjects, 18 (56.25%) were males, and 14 (43.75%) were females. Only 30 teeth were evaluated after six months. Twenty-seven restorations were evaluated as successful while three were evaluated as a failure, which gives a 90% survival rate. Restorations considered to have survived are scored by code: 0,1,7; those considered to have failed by code: 2,3,4,8; while those that are considered to be unrelated to success and failure are scored by code: 5,6. Out of 30 teeth, 22 restored teeth were present in good condition when evaluated after six months, while one tooth showed a gross defect of more than 1.0 mm in depth where the repair was required and two teeth showed complete loss of restoration as examined by the professional dentist. After the ART procedure, microbiological assessment of salivary Streptococcus mutans showed a reduction in the colony-forming units from baseline to six months (Table 3).

**Table 3:** CFU of SM at several time intervals CFU: Colony forming units; SM: Streptococcus mutans

Colony forming units (CFU) intervals	N	Mean	Std. Deviation	Minimum	Maximum
Baseline	32	48.30 x 10^3^	46.58	2.0 x 10^3^	222 x 10^3^
1 week	32	32.64 x 10^3^	30.40	0.9 x 10^3^	122 x 10^3^
1 month	30	18.6 x 10^3^	20.81	0.3 x 10^3^	88 x 10^3^
3 months	30	13.6 x 10^3^	18.04	0.1 x 10^3^	85 x 10^3^
6 months	30	16.2 x 10^3^	23.34	0.3 x 10^3^	120 x 10^3^

At baseline, the mean CFU was 48.30 ± 46.58, which reduced to 32.64 ± 30.40 at one week study period, which showed a 32% reduction in colony counts. A statistically significant difference was seen between baseline CFU and one-week CFU of Streptococcus mutans. One week mean CFU was 32.64 ± 30.40, which reduced to 18.60 ± 20.81 at one month study period, which showed a 43% reduction in colony counts. A statistically significant difference was observed between one-week CFU and one-month CFU of Streptococcus mutans. At one month, the mean CFU was 18.60 ± 20.81, which reduced to 13.63 ± 18.04 in three months study period, which showed a 27% reduction in colony counts. The difference observed was statistically significant between one month and three months CFU of Streptococcus mutans. Three-month mean CFU was 13.63 ± 18.04, which increased to 16.23 ± 23.34 during six months study period, which showed a 19% increase in colony counts. The difference observed was statistically significant between three months and six months CFU of Streptococcus mutans. Comparison of baseline mean CFU (48.30 ± 46.58) to six months mean CFU of Streptococcus mutans (16.23 ± 23.34) showed a 66% reduction in colony counts difference was statistically significant (Table 4).

**Table 4:** Comparison of mean CFU of SM at various time intervals % - Percentage; S - Significant; CFU: Colony forming units; SM: Streptococcus mutans p<0.05 statistically significant.

	Baseline	1 week	Baseline-1 week	1 month	1 week-1 month	3 months	1 month-3 months	6 M	3 months-6 months	Baseline-6 months
Mean	48.30	32.64	15.68	18.60	14.04	13.63	4.97	16.23	-2.6	41.09
Std. Deviation	46.58	30.40	-	20.81	-	18.04	-	23.34	-	-
% Reduction	-	-	32	-	43	-	27	-	19	66
Range	2-222	.9-122	-	.3-88	-	.1-85	-	.3-120	-	-
Z-value	-	-	4.937	-	4.782	-	4.618	-	3.734	4.783
p-value	-	-	0.001 (S)	-	0.001 (S)	-	0.001 (S)	-	0.001 (S)	0.001 (S)

## Discussion

Dental caries is a public health concern in India, with prevalence rates ranging from 50% to 85%. For lessening disease prevalence and severity, a need for alternative treatment methods rather than conventional restorative treatment is required. Given the difficulty of providing oral care to such a large population, the ART approach, which does not necessitate specialized and expensive dental equipment, may be the best option. Several studies have been conducted on the ART technique [11-14], which has produced satisfactory restoration success for up to three years. The success rate is higher for the restoration of permanent teeth than for primary teeth. Only a few studies revealed a significant reduction in salivary SM after an ART restoration. Owing to their metabolic features and activity, the mutans group of streptococci is widely recognized as the most cariogenic bacterium. However, effective treatment to counteract this confounding factor, whether from carious lesions or the entire oral cavity, has always been difficult for the dentistry profession, as no effective treatment to completely eliminate it from the oral cavity exists [15].

For our study, ART was performed on 32 permanent teeth and evaluated after six months. Pre-treatment counts of salivary Streptococcus mutans in the sample size of 32 children displayed raised reflection of disease severity, which was in agreement with Songpaisan et al. [16]. Our data displayed a significant decline in Streptococcus mutans count in one week (32%), one month (43%), three months (27%), and six months (66%) after ART. After ART, there was a statistically significant reduction from baseline to six months period. The results displayed Streptococcus mutans levels to be reduced significantly immediately following one week in 96% of children with mean CFUs reduced from baseline (48.30 x 10^3^) to one week with CFUs of 32.64 x 10^3^. This agrees with other research by Carvalho and Bezerra [5], Ersin et al. [17], and Frencken et al. [18]. More recent studies include Sherief et al. [19] and Hesse et al. [20] in 2020 and 2021, respectively. This is explained by the report that suggests glass ionomer cement (GIC) possesses an antibacterial property owing to fluoride release that also potentiates remineralization [21,22].

A significant reduction in the mean CFU of Streptococcus mutans up to three months after the ART could be due to the antibacterial effect of GIC cement and fluoride release, which is proved in many in vitro and in vivo studies. The children who received treatment also received a health education program regarding brushing habits, and along with this, dietary counseling was also done. Our study displayed a reduction in SM count observed throughout the study period of six months which was contrary to other studies reported by Carvalho and Bezerra [5] where the reduction was marked till one year. This was mainly due to the inclusion of topical fluoride application every six months during the study period. The children who participated also received fluoridated toothpaste, and it is essential to underline that all participants were born and raised in fluoridated environments. All of these fluoride sources have been shown in previous research to aid fluoride uptake by GIC restorations. This effect could have impacted the drop in SM levels after a year. Previous studies have stated that prolonged fluoride release is due to a principal characteristic of GIC (FUJI IX), its potential to recharge fluoride by applying acidulated phosphate fluoride (APF) gel, NaF, and is influenced by pH and concentration of recharge agent. The mechanism of fluoride in recharge is still unclear. It may occur partly by the washout of remnants of viscous gel from pores and cracks in materials or partly by erosion of their surfaces in the presence of low pH agents or by diffusion of fluoride ions taken up by restorative matrix [23].

The microbial levels in our study decreased with ART treatment but increased three months after the treatment. This result is in accordance with Keene et al. [24]. However, one explanation for the resurgence of Streptococcus mutans could be attributed to the organism’s ability to colonize the restored surfaces readily. Our data indicate that the association between caries and SM counts would not be exact in all of the cases studied. The testing for this bacteria is still useful as a predictor of future dental caries as reported by Bowden [25].

Using the ART procedure, it is not impossible to maintain salivary Streptococcus mutans numbers at lower levels. It is crucial to highlight that these mechanical techniques, in combination with infection control achieved by removing carious tissue and bacteria, could have had both qualitative and quantitative effects on bacterial counts, influencing the results. The use of glass ionomer cement and the provision of health education to all children may have led to a sustained reduction in counts that was visible after six months. All through the six-month study period following ART, the SM count in saliva showed a substantial decrease. Because of the limited numbers, the study's potential to detect change was low, and more thorough research is needed before solid conclusions can be formed. Although the above results are required to be conﬁrmed for a larger and more stratified population with the details of their preventive configurations to combat this multifactorial disease. For future implications, it is essential to be evaluated in a larger population considering other clinical parameters pertaining to dental caries development.

## Conclusions

ART is a technique that can be used to provide restorative dental care to young children outside of a typical clinic environment. It is highly appropriate, effective, and acceptable. Adopting the ART technique in dental outreach initiatives in the school setting can assist enhance access to dental care in most developing countries because it is not reliant on expensive and complex dental equipment. The data show that ART is an effective clinical procedure for treating caries in young children, as well as a method for lowering SM levels in saliva. Nevertheless, more research is needed, particularly in field trials, to a better scientific understanding of when and how to employ the procedure.

## References

[1] (2020). WHO Oral Health (1994). http://www.who.int/aboutwho/en/promoting/oral.htm.

[2] (2020). WHO Oral Health Activities (2002). http://www.who.int/ncd/orh/orh_act.htm.

[3] WHO. (28 - 7 April 1994 (2020). WHO. Revolutionary new procedure for treating dental caries. http://www.who.int/archieves/inf-pr-1994/pr94-28.htm.

[4] World Health Organization (2020). Manual - Técnica de Restauración Atraumatica Para El Tratamiento de la Dental Caries. http://www.bvsops.org.uy/pdf/uru76.pdf.

[5] Carvalho CKS, Bezerra ACB (2003). Microbiological assessment of saliva from children subsequent to atraumatic restorative treatment (ART). Int J Paediatr Dent.

[6] Bönecker M, Toi C, Cleaton-Jones P (2003). Mutans streptococci and lactobacilli in carious dentine before and after atraumatic restorative treatment. J Dent.

[7] van Houte J (1994). Role of micro-organisms in caries etiology. J Dent Res.

[8] Loesche WJ, Syed SA (1973). The predominant cultivable flora of carious plaque and carious dentine. Caries Res.

[9] Frencken JE, Songpaisan Y, Phantumvanit P, Pilot T (1994). An atraumatic restorative treatment (ART) technique: evaluation after one year. Int Dent J.

[10] Emilson CG, Krasse B (1986). Comparison between a dip-slide test and plate count for determination of Streptococcus mutans infection. Scand J Dent Res.

[11] Phantumvanit P, Songpaisan Y, Pilot T, Frencken JE (1996). Atraumatic restorative treatment (ART): a three-year community field trial in Thailand--Survival of one-surface restorations in the permanent dentition. J Public Health Dent.

[12] Frencken JE, Makoni F, Sithole WD (1998). ART restorations and glass ionomer sealants in Zimbabwe: survival after 3 years. Community Dent Oral Epidemiol.

[13] Holmgren CJ, Lo EC, Hu D, Wan H (2000). ART restorations and sealants placed in Chinese school children--results after three years. Community Dent Oral Epidemiol.

[14] Lopez N, Simpser-Rafalin S, Berthold P (2005). Atraumatic restorative treatment for prevention and treatment of caries in an underserved community. Am J Public Health.

[15] Keene HJ, Shklair IL, Hoerman KC (1976). Partial elimination of Streptococcus mutans from selected tooth surfaces after restoration of carious lesions and SnF2 prophylaxis. J Am Dent Assoc.

[16] Songpaisan Y, Serinirach R, Kuvatanasuchati J, Bratthall D (1994). Mutans streptococci in a Thai population: relation to caries and changes in prevalence after application of fissure sealants. Caries Res.

[17] Ersin NK, Uzel A, Aykut A, Candan U, Eronat C (2006). Inhibition of cultivable bacteria by chlorhexidine treatment of dentin lesions treated with the ART technique. Caries Res.

[18] Frencken JE, Imazato S, Toi C, Mulder J, Mickenautsch S, Takahashi Y, Ebisu S (2007). Antibacterial effect of chlorhexidine-containing glass ionomer cement in vivo: a pilot study. Caries Res.

[19] Sherief DI, Fathi MS, Abou El Fadl RK (2021). Antimicrobial properties, compressive strength and fluoride release capacity of essential oil-modified glass ionomer cements-an in vitro study. Clin Oral Investig.

[20] Hesse D, Guglielmi CA, Raggio DP, Bönecker MJ, Mendes FM, Bonifácio CC (2021). Atraumatic restorative treatment-sealed versus nonsealed first permanent molars: a 3-year split-mouth clinical trial. Caries Res.

[21] Malik S, Ahmed MA, Choudhry Z, Mughal N, Amin M, Lone MA (2018). Fluoride release from glass ionomer cement containing fluoroapatite and hydroxyapatite. J Ayub Med Coll Abbottabad.

[22] Mukai M, Ikeda M, Yanagihara T, Hara G, Kato K, Nakagaki H, Robinson C (1993). Fluoride uptake in human dentine from glass-ionomer cement in vivo. Arch Oral Biol.

[23] Yip HK, Smales RJ (2000). Fluoride release from a polyacid-modified resin composite and 3 resin-modified glass-ionomer materials. Quintessence Int.

[24] Keene HJ, Shklair IL, Mickel GJ (1977). Effect of multiple dental floss-SnF2 treatment on Streptococcus mutans in interproximal plaque. J Dent Res.

[25] Bowden GH (1996). Mutans streptococci caries and chlorhexidine. J Can Dent Assoc.

